This article has been retracted.

# miR-215 Inhibits Colorectal Cancer Cell Migration and Invasion via Targeting Stearoyl-CoA Desaturase

**DOI:** 10.1155/2020/5807836

**Published:** 2020-06-30

**Authors:** Xinhua Xu, Yan Ding, Jun Yao, Zhiping Wei, Haipeng Jin, Chen Chen, Jun Feng, Rongbiao Ying

**Affiliations:** ^1^Department of Pathology, Taizhou Cancer Hospital, Zhejiang Province, China; ^2^Department of Radiotherapy Oncology, Taizhou Central Hospital, Zhejiang Province, China; ^3^Department of Surgical Oncology, Taizhou Cancer Hospital, Zhejiang Province, China

## Abstract

**Background:**

This study was aimed at exploring the effects of miR-215 and its target gene stearoyl-CoA desaturase (SCD) on colorectal cancer (CRC) cell migration and invasion.

**Methods:**

Here, we analyzed the relationship between miR-215 and SCD, as well as the regulation of miR-215 on CRC cells. We constructed wild-type and mutant plasmids of SCD to identify whether SCD was a target gene of miR-215 by using a luciferase reporter assay. The expression of miR-215 and SCD was detected by quantitative real-time polymerase chain reaction (qRT-PCR) and western blot, respectively. MTT, wound healing, and Transwell assays were applied to determine the effect of miR-215 on CRC cell proliferation, migration, and invasion.

**Results:**

It was found that miR-215 expression was significantly decreased in CRC tissue while SCD was highly expressed compared with those in adjacent normal tissue. The luciferase reporter assay indicated that SCD was a direct target gene of miR-215. Functional analysis revealed that miR-215 overexpression significantly inhibited CRC cell proliferation, migration, and invasion *in vitro*. In addition, the result of rescue experiments showed that overexpression of SCD could promote the proliferation, migration, and invasion of CRC cells, and the carcinogenic effect of SCD could be inhibited by miR-215.

**Conclusions:**

Taken together, our findings suggested that miR-215 could inhibit CRC cell migration and invasion via targeting SCD. The result could eventually contribute to the treatment for CRC.

## 1. Background

Colorectal cancer (CRC) is one of the common malignant cancers of the digestive tract, including the rectum and colon, which mainly occurs in the rectum and the junction between the rectum and sigmoid colon. CRC is also the third most frequently diagnosed cancer and the fourth leading cause of cancer-related death globally [1, 2]. Although cancer treatment strategies are increasingly developed and the treatment effect of CRC patients in early stages has been significantly improved during the past several decades, most patients have been already diagnosed in advanced stages. At present, surgical resection is the most effective method of treating CRC, but 25%-40% of patients still experience recurrence or metastasis. Therefore, it has become a hot topic to explore the invasion and migration of CRC cells at the molecular level, which helps to find new effective treatment options and improve patients' survival rate.

Stearoyl-CoA desaturase (SCD) is a key enzyme for the formation of monounsaturated fatty acids from saturated fatty acids, and its main components include palmitoleic acid (C16:1) and oleic acid (C18:1) [3]. In recent years, SCD has been confirmed to play an important regulatory role in the occurrence and development of a variety of cancers. For example, decreased SCD expression can inhibit breast cancer progression through the *β*-catenin signaling pathway [4]. SCD can significantly promote the growth of lung cancer by activating EGFR/PI3K/AKT signaling in tumor tissue [5]. However, the regulatory mechanism of SCD in CRC remains unclear.

MicroRNAs (miRNAs) are a class of small noncoding RNAs that can regulate gene expression by facilitating mRNA degradation or inducing translational repression [6]. The miRNA miR-215 has been proven to play an important role in tumorigenesis and tumor progression in many types of human cancers, such as epithelial ovarian cancer (EOC) [7], endometrial cancer [8], breast cancer [9], and non-small-cell lung cancer [10]. Recent studies show that overexpression of miR-215 markedly downregulates LEFTY2 protein expression level in HEc-1A cells and endometrial cancer tissue [11]. It is also reported that overexpression of LEFTY2 protein promotes epithelial-mesenchymal transition (EMT) and sensitizes HEc-1A cells to cisplatin treatment [11]. In addition, overexpression of miR-215 suppresses EOC growth and invasion by targeting NOB1 [12]. However, the relationship between miR-215 and SCD has not been reported yet.

In this study, we tested miR-215 expression in CRC cells and investigated the biological effect of miR-215 on migration and invasion of CRC cells. Here, we found that miR-215 exerted a suppressive effect on tumor migration and invasion by targeting SCD.

## 2. Methods

### 2.1. Microarray Analysis

We searched the Gene Expression Omnibus (GEO) database (https://www.ncbi.nlm.nih.gov/geo/) with “Colorectal cancer” as the key word, and two miRNA microarrays GSE110224 and GSE35834 were selected. GSE110224 included 17 normal samples and 17 tumor samples with histologically confirmed CRC. Total mRNAs were extracted for further processing with the Human Genome U133 Plus 2.0 Array (Affymetrix Inc., Santa Clara, CA, USA). GSE35834 contained 78 samples comprising 23 normal adjacent mucosa tissue samples and 55 CRC tumor samples, and GPL8786 Multispecies miRNA-1 Array (Affymetrix Inc., Santa Clara, CA, USA) was used as the sequencing platform. The datasets were analyzed with the R package “Limma.” ∣logFC | >1 and *p* value < 0.05 were set as the threshold for screening the differentially expressed genes (DEGs).

### 2.2. Analysis of the miRNAs That Regulate SCD

The miRNAs that regulate SCD were retrieved in the starBase V2.0 (http://starbase.sysu.edu.cn/), TargetScan (http://www.targetscan.org/), and miRTarBase (http://mirtarbase.mbc.nctu.edu.tw/) databases. A Venn diagram (http://bioinformatics.psb.ugent.be/webtools/Venn/) was used to find the intersections of the predicted results in the three databases.

### 2.3. Human Tissue Specimens

Paraffin-embedded pathological specimens from 30 CRC tumor and paired adjacent normal tissue samples were included in this study. Samples were obtained from Taizhou Cancer Hospital, Zhejiang Province, from July 2016 to June 2017. All the patients were diagnosed by pathological examination and had never received chemotherapy or radiotherapy before surgery. All the samples were collected with patients' informed consent after approval from the Institute Research Medical Ethics Committee of Taizhou Cancer Hospital.

### 2.4. Cell Lines and Transfection

The CRC cell line HT29 was obtained from the Bena Culture Collection (Beijing, China) and was grown in Dulbecco's Modified Eagle's Medium (DMEM, Gibco) with 100 U/mL penicillin, 0.1 mg/mL streptomycin, and 10% fetal bovine serum (FBS). All cells were maintained in a humidified incubator with 5% CO_2_ at 37°C until they were grown to a logarithmic phase. Cells (2 × 10^5^ cells/well) were seeded in a six-well plate and then subjected to transfection by employing Lipofectamine 2000 (Invitrogen, Karlsruhe, Germany).

NC (transfected with negative sequence), miR-215 mimic, and miR-215 inhibitor were purchased from GeneCopoeia (Guangzhou, China). SCD overexpression (oe-SCD) and corresponding negative control (oe-NC) were constructed by lentiviral vectors.

### 2.5. Dual-Luciferase Reporter Gene Assay

Target sequences of wild-type (WT) and mutant (WUT) SCD 3′UTR were constructed artificially and ligated into the pmirGLO (Promega, Madison, USA) reporter plasmids with enzymes BamHI and XhoIII to obtain WT and MUT reporter plasmids. Afterwards, the two reporter plasmids were cotransfected with the miR-215 mimic or NC into the cancer cell line using Lipofectamine 2000. Relative luciferase activities were determined by the Dual-Luciferase® Reporter Assay System (Promega) following the instructions 48 h after transfection.

### 2.6. qRT-PCR

Total RNA was extracted from CRC cells, tumor tissue, and paired adjacent normal tissue using Trizol Reagent (Ambion, USA) according to the manufacturer's instructions. The concentration and purity of RNA were determined with an ultraviolet spectrophotometer. RNA was reversely transcribed into cDNA by using RT-PCR Kit (ABI Company, 243 Forest City, CA, USA), and quantitative real-time- (qRT-) PCR was performed according to the manufacturer's instructions of SYBR Premix Ex Taq II (TaKaRa). The relative expression level of RNA was calculated by the 2^-*ΔΔ*CT^ method with U6 and GAPDH as the internal reference for miR-215 and SCD, respectively. miR-215 stem-loop primers were as follows: 5′-CTCAACTGGTGTCGTGGAGTCGGCAATTCAGTTGAGCGTCTGT-3′. The sequences of the PCR primers were as follows: miR-215 forward 5′-CTCAACTGGTGTCGTGGAGTCGG-3′ and reverse 5′-ACAGGAAAATGACCTATGAATTGAC-3′, U6 forward 5′-GTACAAAATACGTGACGTAGAAAG-3 and reverse 5′-GGTGTTTCGTCCTTTCCAC-3′, SCD forward 5′-TCTAGCTCCTATACCACCACCA-3′ and reverse 5′-TCGTCTCCAACTTATCTCCTCC-3′, and GADPH forward 5′-GGAGCGAGATCCCTCCAAAAT-3′ and reverse 5′-GGCTGTTGTCATACTTCTCATGG-3′.

### 2.7. Western Blot Analysis

Cells in the logarithmic growth phase were collected and lysed with the RIPA buffer containing protease and phosphatase inhibitors. Extracted proteins were loaded onto 8% SDS-PAGE at a voltage of 150 V after quantification. Thereafter, the proteins were transferred onto the PVDF membrane and incubated with the primary mouse antibodies against SCD (1 : 500, Abcam) and GADPH (1 : 1000, Abcam), respectively, overnight at 4°C. After three times being washed with TBST, the membrane was probed with the secondary antibody rabbit anti-mouse IgG (HRP) (1 : 2000, Abcam) for 1 h at room temperature. Finally, the protein bands were detected using the ABI 7500 Real-Time PCR System (Applied Biosystems; Thermo Fisher Scientific, NY, USA).

### 2.8. MTT

The MTT assay was conducted to evaluate cell proliferation capacity. Cells were trypsinized after 24 h of culture in serum-free medium. The cells were counted with a hemocytometer, and the cell density was adjusted to 1 × 10^5^ cells/mL. Then, the cells were seeded in 96-well plates at a density of 2 × 10^3^ cells/well with the volume of 200 *μ*L. 5 mg/mL of MTT solution was added to each well at 24 h, 48 h, and 72 h, respectively. After incubation for 4 h, the reaction was stopped. The supernatant was discarded after centrifugation, and 100 *μ*L of DMSO was added to each well to promote crystal dissolution. The absorbance was measured at 490 nm. The assay was performed in triplicate.

### 2.9. Wound Healing Assay

CRC cells in the logarithmic phase were inoculated into a 6-well plate (2 × 10^5^ cells/well) with marks on the back of the plate. After 24 h of culture, the cells covered the entire plate, and scratches were created perpendicular to the marks using a 10 *μ*L pipette. The detached cells were washed away with PBS, followed by the addition of serum-free DMEM. Cells were incubated in an incubator with 5% CO_2_ at 37°C, and images at 0 h and 48 h were captured under an inverted microscope. Three parallel wells were prepared for each group.

### 2.10. Transwell Invasion Assay

Transwell inserts (Millipore, Bedford, Mass., USA) covered with Matrigel were used for a cell invasion assay. CRC cells in the logarithmic phase were harvested for digestion with trypsin, then washed once with PBS and resuspended in serum-free DMEM. The cell density was adjusted to 1 × 10^5^ cells/mL. A total of 200 *μ*L of cell suspension was seeded in the upper chambers, and 500 *μ*L of DMEM containing 15% FBS was added to the lower chambers. The cells were then cultured in an incubator with 5% CO_2_ at 37°C for 48 h. Cells invading the lower chambers were fixed with 95% ethanol for 10 min and stained with 0.1% crystal violet for 10 min, and PBS was used to remove the unstained cells. After observation under an inverted microscope, cells from 5 randomly selected fields were counted and the mean value was determined. This experiment was repeated three times. The number of cells that penetrated the Matrigel showed the invasion ability of cells in each group.

### 2.11. Statistical Analysis

Statistical analysis was conducted using SPSS 21.0 software and GraphPad Prism 6.0. Experiment data were recorded as the mean ± standard deviation. Comparisons between two groups were assessed by Student's *t*-test, while comparisons among multiple groups were assessed by one-way ANOVA. Counting data were analyzed by the chi-square test. *P* < 0.05 was considered statistically significant.

## 3. Results

### 3.1. SCD Is Upregulated in CRC

The transcriptome expression data of CRC were analyzed by the bioinformatics method. The results showed that SCD was significantly upregulated in CRC samples compared with normal samples (Figures 1(a) and 1(b)). At the same time, the qRT-PCR result showed that the expression level of SCD mRNA in CRC tissue was significantly higher than that in adjacent tissue (Figure 1(c)).

### 3.2. SCD Is a Direct Target Gene of miR-215

In order to explore the underlying mechanism of SCD in CRC cells, we firstly analyzed the GSE35834 dataset and obtained 20 miRNAs with significant differential expression in CRC (Figure 2(a)). Then, the starBase V2.0, TargetScan, and miRTarBase databases were used to predict the potential upstream miRNAs for SCD (Figure 2(b)). According to bioinformatics databases, there was a binding site of miR-215 and 3′-UTR of SCD (Figure 2(c)). In addition, the expression level of miR-215 in CRC tissue was significantly decreased (Figure 2(d)).

To confirm whether SCD was a direct target gene of miR-215 in CRC cells, we conducted the luciferase reporter assay in HT29 cells 48 h after cotransfection of WT or MUT SCD and miR-215 mimic or NC. The result exhibited that overexpression of miR-215 reduced the luciferase activity of WT SCD in HT29 cells but had no effect on MUT SCD (Figure 2(e)). Additionally, overexpression of miR-215 significantly inhibited the mRNA and protein expression of SCD (Figures 2(f) and 2(g)). Subsequently, we analyzed the correlation between miR-215 and SCD expression in clinical specimens. The result indicated that there was a negative correlation between them (Figure 2(h)). These results indicated that SCD was a direct target gene of miR-215.

### 3.3. miR-215 Inhibits CRC Cell Proliferation, Migration, and Invasion *In Vitro*

According to the aberrant expression of miR-215 in CRC cells, we speculated that it might regulate cancer cell proliferation, invasion, and migration. In order to test our hypothesis, we overexpressed and inhibited miR-215 in HT29 cells by transfecting the miR-215 mimic and inhibitor, respectively. qRT-PCR was used to confirm that the miR-215 expression was decreased significantly in the miR-215 inhibitor group and increased in the miR-215 mimic group (Figure 3(a)). After transfection, we used the MTT assay to evaluate the cell proliferation capacity at 24 h, 48 h, and 72 h. The result observed low proliferation activity of HT29 cells after overexpressing miR-215 (Figure 3(b)). Meanwhile, we investigated whether miR-215 affected CRC cell invasion and migration. Wound healing and Transwell invasion assays were performed in HT29 cells transfected with NC, miR-215 mimic, and miR-215 inhibitor. The results demonstrated that overexpression of miR-215 significantly inhibited cell invasion and migration (Figures 3(c) and 3(d)).

### 3.4. miR-215 Mediates the Migration and Invasion of CRC Cells via Targeting SCD

In order to verify that miR-215 can regulate the cellular function of CRC cells by inhibiting the expression of SCD, we conducted the rescue experiments. Firstly, we detected the mRNA and protein levels of SCD in three transfected HT29 cell lines (NC+oe-NC, NC+oe-SCD, and miR-215 mimic+oe-SCD), and the results showed that the elevated expression of SCD was downregulated by miR-215 (Figures 4(a) and 4(b)). Then, we measured the proliferation of cancer cells through the MTT assay and discovered that overexpression of SCD promoted the proliferation of cancer cells, and its promoting effect could be reversed by overexpression of miR-215 (Figure 4(c)). In addition, we used the wound healing assay and Transwell invasion assay to detect the migration and invasion of cells. The results indicated that the overexpression of SCD significantly promoted the migration and invasion of HT29 cells, while the simultaneous overexpression of miR-215 and SCD attenuated such promoting effect (Figures 4(d) and 4(e)). Therefore, we believed that miR-215 could inhibit the proliferation and migration of CRC by downregulating the expression of SCD.

## 4. Discussion

More than 1.2 million patients are diagnosed with CRC each year. The mortality of CRC is the fourth highest of all the cancer deaths, and the disease tends to be younger in epidemiology. Therefore, studying the mechanism of occurrence, invasion, and migration of CRC can improve the therapeutic effect of CRC patients. Accumulating evidence shows that miRNAs are closely related to the proliferation, invasion, migration, and recurrence of various tumors, and they can be used as effective molecular markers as well as therapeutic targets for cancer diagnosis, prognosis, and treatment [13–15].

In this study, we found that SCD was highly expressed in CRC by bioinformatics. The literature on SCD has also showed that SCD is upregulated in multiple cancers, such as ovarian cancer [16], breast cancer [17], and liver cancer [18]. Next, in order to verify the result of bioinformatics, we detected the expression of SCD in normal tissue and CRC tissue and confirmed that SCD was upregulated in CRC tissue. It is universally known that miRNAs exert their biological functions by regulating the expression of target genes [19]. Therefore, we used bioinformatics to further explore the miRNAs that could target SCD, and it was found that miR-215 and SCD had binding sites. miR-215 is a widely studied miRNA that has been confirmed to targetedly inhibit various mRNAs, including ARFGEF1 [20], RUNX1 [21], KDM1B [22], and ZEB2 [10]. In order to verify that SCD was a downstream target of miR-215, we detected the expression of miR-215 in normal tissue and CRC tissue by qRT-PCR and found that miR-215 was downregulated in CRC, and the expression of miR-215 was negatively correlated with SCD expression in CRC tissue. Meanwhile, the dual-luciferase assay verified the binding sites of miR-215 on SCD. In addition, we detected the expression of SCD after overexpressing miR-215 in CRC cells, and it was also discovered that miR-215 could inhibit the expression of SCD in CRC cells. Thus, SCD was fully confirmed to be a downstream target of miR-215. Published literature indicates that the dysregulated miRNAs and mRNAs may have the function of regulating the occurrence and development of CRC [23–25]. Therefore, we further observed the effect of miR-215 on the proliferation, migration, and invasion of CRC cells through MTT, wound healing, and Transwell invasion assays and found that miR-215 had a significant inhibitory effect on CRC cells, while SCD could attenuate the inhibitory effect of miR-215 on CRC cells. The above results suggested that miR-215 could inhibit the proliferation, migration, and invasion of CRC cells by targeting SCD.

In summary, we demonstrated that the expression of miR-215 was downregulated in CRC tissue compared with adjacent normal colorectal tissue. miR-215 impaired CRC cell proliferation, migration, and invasion *in vitro* by inhibiting the expression of SCD. The results of this study contribute to the improvement of the understanding of the molecular mechanism underlying CRC development and progression and provide potential new therapeutic targets for the management of CRC.

## Figures and Tables

**Figure 1:** SCD is upregulated in CRC, and the number unit is expression log_2_. (a) The top 20 DEGs in GSE110224. (b) The SCD gene is significantly upregulated in CRC samples. (c) qRT-PCR is used to detect the expression of the SCD gene in cancer tissue and paracancerous tissue (*n* = 30, ^∗^*P* < 0.05).

**Figure 2:** SCD is a direct target gene of miR-215. (a) The top 20 DEmiRNAs in GSE35834. (b) The Venn diagram of miRNAs that regulate SCD. (c) The targeting sites of miR-215 on SCD 3′UTR and the corresponding mutant sequences. (d) qRT-PCR is used to detect the expression of miR-215 in cancer tissue and paracancerous tissue (*n* = 30, ^∗^*P* < 0.05). (e) Relative luciferase activity in HT29 cells after cotransfection with WT or MUT SCD and miR-215 mimic or NC (^∗^*P* < 0.05, ^∗∗^*P* < 0.01, compared to NC). (f) SCD expression on mRNA level in HT29 cells transfected with the miR-215 mimic or NC (^∗^*P* < 0.05, compared to NC). (g) SCD expression on the protein level in HT29 cells transfected with the miR-215 mimic or NC. (h) The correlation between miR-215 and SCD expression in clinical specimens (^∗^*P* < 0.05, compared to NC).

**Figure 3:** miR-215 inhibits CRC cell proliferation, invasion, and migration *in vitro*. (a) qRT-PCR is used to confirm the transfection efficiency of miR-215. (b) Cell proliferation is determined by the MTT assay. (c) Cell migration is determined by the wound healing assay. (d) The invasion of HT29 cells is examined using the Transwell assay, and the representative images are presented (^∗^*P* < 0.05, compared to NC).

**Figure 4:** miR-215 mediates the proliferation, migration, and invasion of CRC cells by targeting SCD. (a) SCD mRNA expression is measured by qRT-PCR. (b) SCD protein expression is detected by western blot. (c) Cell proliferation is determined by the MTT assay. (d) Cell migration is examined by the wound healing assay. (e) The invasion of HT29 cells is examined using the Transwell assay, and the representative images are presented (^#^*P* < 0.05, compared to NC+oe-NC; ^∗^*P* < 0.05, compared to NC+oe-SCD; NC is the control of the miR-215 mimic, and oe-NC is the control of oe-SCD).

## Data Availability

The data used to support the findings of this study are available from the corresponding author upon request.
